# Study on Influencing Factors of Radial Artery Occlusion after Repeated Right Radial Artery Coronary Intervention

**DOI:** 10.1155/2022/9624339

**Published:** 2022-07-16

**Authors:** Jianbing Wang, Chunxue Yi, Jianming Zhang

**Affiliations:** Cardiovascular Department of Chongqing University Three Gorges Hospital, Chongqing, China

## Abstract

**Objective:**

To investigate the risk factors of radial artery obstruction after repeated right radial coronary interventions.

**Methods:**

497 patients who underwent repeated coronary intervention via the right radial artery in our hospital from January 2017 to January 2021 were selected and followed up for 28.07 ± 6.07 months. According to whether the right radial artery was obstructed or not, they were divided into radial artery occlusion group (*n* = 48) and nonradial artery occlusion group (*n* = 449).

**Results:**

The proportion of patients with diabetes mellitus, elevated D-dimer, and elevated LDL cholesterol was higher in the radial artery occlusion group than in the nonradial artery occlusion group (*p* < 0.05). The radial artery occlusion group had more passage through the right radial artery often and had a longer cumulative sheath retention time than the radial artery occlusion group (*p* < 0.05). Cumulative sheath retention time (hours) had a high predictive value for radial artery occlusion. The optimal diagnostic limit for radial artery occlusion was 2.75 h, with a sensitivity of 77.1% and a specificity of 79.5% (*p* < 0.05).

**Conclusion:**

Diabetes mellitus, elevated D-dimer, elevated LDL cholesterol, and long retention sheath time predispose to radial artery occlusion. Cumulative duration of sheath retention is a predictor of radial artery occlusion.

## 1. Introduction

The total number of interventional therapies for coronary heart disease in mainland China in 2018 was 915256 based on the report of China Cardiovascular Health and Disease 2020 [1]. The radial artery pathway is the default path for coronary intervention. Compared with the femoral artery pathway, significant development in patient comfort and reductions in puncture site complications were achieved through less-invasive radial artery access [2–4]. Currently, radial artery occlusion is a frequent complication of radial artery access, and it has been reported that radial artery occlusion incidence after coronary intervention was 2% to 10% [5, 6]. The main blood supply of the hand comes from the radial artery and ulnar artery. After radial artery occlusion, the ulnar artery can provide a single blood supply for the hand, so radial artery occlusion is usually asymptomatic in clinic. A repeat coronary intervention was received through the right radial artery in our hospital. The mean follow-up rate was 28.07 ± 6.07 months. A total of 48 cases developed right radial artery occlusion (incidence of 9.66%). The patients are likely to need to undergo coronary artery treatment several times during their lifetime. The radial artery occlusion risk is likely to be enhanced by repeated ipsilateral radial artery punctures. Once the radial artery is occluded, it will lower the likelihood of patients experiencing radial artery intervention again and increase the proportion of femoral artery puncture. Diabetes mellitus, elevated D-dimer, elevated LDL cholesterol, and long retention sheath time predispose to radial artery occlusion. Cumulative duration of sheath retention is a predictor of radial artery occlusion. With long-term follow-up, the aim was to study right radial artery occlusion risk factors after repeat right radial coronary intervention.

## 2. Data and Methods

### 2.1. Study Subjects

We selected 497 patients (356 men and 141 women) as the study population. From January 2017 to January 2021, they received repeat coronary intervention through the right radial artery in our hospital. The average follow-up was 28.07 ± 6.07 months. A total of 48 cases had right radial artery occlusion (the incidence rate was 9.66%). Inclusion criteria included the following: (1) have indications for coronary intervention, complete coronary intervention through the right radial artery at least twice or more in our hospital during the follow-up period, and regularly take dual antiplatelet and statins to reduce blood lipid; (2) no history of macrovascular abnormalities and arteriovenous short circuit in renal dialysis. Exclusion criteria were the following: (1) previous history of interventional diagnosis and treatment via the right radial artery; (2) Allen [7] test abnormality and inverse Allen test abnormality. The symptoms of radial artery occlusion include pain, pallor, syncope, numbness, dyskinesia, and diminished and absent arterial pulsations in the area of blood supply. The severity of symptoms depends on the severity of the occlusion, the amount of secondary thrombosis, the presence of previous atherosclerotic disease leading to arterial stenosis, and the presence of collateral circulation. When radial artery occlusion occurs, the cause should be actively sought and treated to avoid further aggravation of radial artery occlusion, which may cause other arterial stenosis or occlusion. Common causes of radial artery occlusion include thin radial artery, long duration of surgery, intraoperative radial artery thrombosis, and excessive postoperative hemostasis compression.

### 2.2. Research Methods

After the puncture method was disinfected, the right radial artery puncture was routinely adopted during the operation and the bilateral radial artery puncture was adopted for some complex operations. Seldinger's method was used for arterial puncture, and 6F radial artery sheath (Terumo Company, Japan) was inserted. After success, nitroglycerin 100 *μ*g and Lidocaine 20 mg were routinely injected through the sheath to prevent arterial spasm. The sheath was pulled out immediately after operation. After pulling out the sheath, it was wrapped with elastic bandage for 3 hours.

### 2.3. Judgment of Radial Artery Occlusion

The judgment time is one year after the last right radial artery route administration. The radial artery occlusion must satisfy both the standards as follows: (1) the radial artery pulsation shall be checked by the interventional specialist to ensure that the radial artery pulsation cannot be touched or the reverse Allen test is abnormal; (2) the radial artery occlusion was confirmed by color Doppler (Philips epic7c with l12-4 probe) in the first meeting condition.

(1) patients who cannot be relieved by medication, or who have frequent angina pectoris (2) patients with coronary angiography, confirmed left main stem lesions with severe three-branch lesions, these patients will die suddenly at any time if they are not bypassed in time, so for patients with two lesions with severe stenosis in important locations that cannot be treated with intervention, even if angina is not obvious but if the left heart function is poor and the ejection fraction is <50% they should be treated surgically. (3) patients who have failed interventional therapy, or patients with recurrent stenosis after coronary artery bypass grafting, (4) heart rupture after myocardial infarction, pericardial tamponade, septal perforation or papillary muscle rupture, mitral valve closure insufficiency, which require emergency surgery or surgery when the systemic condition is stable. 5, after ventricular wall tumor formation, the ventricular wall tumor can be removed and coronary artery bypass can be done at the same time. For patients with ventricular arrhythmias caused by old infarct scars, endocardiotomy can be considered after cardiac electrophysiological examination. 6. Patients with a relatively large area of obsolescence, also known as large infarction, are obsolete without symptoms of angina pectoris, but with left heart insufficiency and ejection fraction in <40% should be operated, mainly depending on the myocardial survival 7, unstable angina and variant angina, the three branches of the coronary artery lesions have been clear, active medical treatment cannot make the symptoms alleviated, and the electrocardiogram shows ischemic changes and myocardial enzymatic changes, suggesting that myocardial ischemia has not been improved, such patients also need to do surgery. 8, diabetic patients, put the stent on diabetic patients, the possibility of restenosis is quite large, the introduction of drug stent is able to solve some problems, but this part of the patients still need to do bypass surgery.

### 2.4. Data Collection

General information of patients included age, gender, height, and weight; high-risk factors causing atherosclerosis such as diabetes, hypertension, and smoking history; the last laboratory examination indicators of the right radial artery route: blood lipid, D-dimer, C-reactive protein, uric acid, and serum creatinine; whether it was emergency coronary intervention at the first visit; the cumulative number of coronary interventions performed; and the cumulative retention time measured through the right radial artery.

### 2.5. Statistical Analysis

SPSS25.0 statistical software is adopted for all statistical analyses. The mean ± standard deviation or median (lower quartile∼upper quartile) represents the measurement data; the *t*-test or nonparametric test (Mann–Whitney *U* test) is used to represent the comparison between the groups of measurement data. The chi square test is selected for the comparison between the counting data groups. Multivariate regression (OR) was used to study the multivariate effect. *p* < 0.05 was considered a difference and was statistically significant.

## 3. Results

### 3.1. Comparison of Baseline Data between the Two Groups

Compared with the nonradial artery occlusion group (*n* = 449), the proportion of patients with diabetes, elevated D-dimer, and elevated low-density lipoprotein cholesterol in the radial artery occlusion group (*n* = 48) was higher, with *p* < 0.05. There was more passage through the right radial artery in the radial artery occlusion group than in the nonradial artery occlusion group. And, the cumulative indwelling sheath time was longer (*p* < 0.05). The differences of other variables were not statistically significant (see Table 1 for details).

### 3.2. Multivariate Analysis

Analysis was performed based on the comparative results of the above baseline data, diabetes mellitus, elevated LDL cholesterol, elevated D-dimer, cumulative time of retention of the right radial artery sheath, and passage through the right radial artery, and further binary logistic regression analysis was performed. The results showed that elevated low-density lipoprotein cholesterol (OR = 3.799, 95% CI (1.292∼11.166), *p*=0.015), diabetes mellitus (OR = 2.186, 95% CI (1.014∼4.714), *p*=0.046), elevated D-dimer (OR = 2.998, 95% CI (1.381∼6.51), *p*=0.006), and accumulated sheath time of the right radial artery (OR = 5.692, 95% CI (3.342∼9.694), *p* < 0.001) were independent risk factors.  Table 2 shows the specific information of right radial artery occlusion.

### 3.3. Diagnostic Value of Accumulated Indwelling Sheath Time (Hours) for Radial Artery Occlusion

The AUC of the ROC curve of cumulative indwelling sheath time (hours) was 0.843 (95% CI 0.778∼0.909). The best diagnostic limit of the radial artery occlusion was 2.75 hours, the sensitivity was 77.1%, and the specificity was 79.5%, with *p* < 0.05 (see Figure 1 for details).

## 4. Discussion

Acute injury and spasm of the intima and middle layer of the radial artery caused by radial artery puncture and indwelling sheath are the main mechanisms of radial artery occlusion. In [8], OCT intervention of the radial artery after radial artery surgery showed that 67.1% of radial arteries had varying degrees of intimal tears after surgery and the incidence of media entrapment was as high as 35.6%. The natural protective barrier of the vasculature is disrupted with the destruction and shedding of vascular endothelial cells. On the one hand, it can activate platelets and the coagulation system to form thrombi and cause acute occlusions. On the other hand, it may lead to endothelium-dependent vasodilatory dysfunction [9]; although lesions tend to heal over time, endothelial integrity and function are still not fully restored [10]. In addition, sheath injury leads to migration of smooth muscle cells into the endothelium, resulting in endothelial-media hyperplasia and increased vessel thickness, which may be an important cause of chronic stenosis or occlusion of the radial artery [11, 12].

With advances in guidewire, sheath, and catheter technology, as well as the utilization of antiplatelet and anticoagulant drugs, the risk of radial artery occlusion within 30 days has decreased to 2–4%. Therefore, a common clinical treatment is repeated coronary intervention through the right radial artery. This study found that the incidence of radial artery occlusion after repeated coronary intervention via the right radial artery was approximately 9.96%, and the multifactorial analysis showed that diabetes mellitus, elevated D-dimer, elevated LDL cholesterol, and the cumulative retention sheath time were high-risk factors for right radial artery occlusion; therefore, effective control of these high-risk factors could effectively prevent radial artery occlusion.

The duration of transradial access and cumulative retention sheath time are an objective reflection of radial artery injury via the radial artery access. The cumulative time was greater in the radial artery occlusion group, and their cumulative retention time was longer than in the nonradial artery occlusion group observed through the right radial artery [13].

In addition, according to Wakeyamat et al. [14], the intima-media thickness after repeated radial artery intervention was studied by using intravascular ultrasound and it was discovered that the intima-media thickness of the radial artery was significantly thickened by the repeated radial artery approach. The conclusion of multivariate analysis for right radial artery occlusion showed that the cumulative indwelling sheath time was an independent risk factor (OR = 5.692, 95% CI (3.342∼9.694), *p* < 0.001). The best diagnostic threshold of cumulative indwelling sheath time for the diagnosis of radial artery occlusion was 2.75 hours; radial artery occlusion risk increased by 5.692 times for each hour of cumulative indwelling sheath time; the AUC of the ROC curve was 0.843 (95% CI 0.778∼0.909) with a sensitivity of 77.1% and a specificity of 79.5%. In this study, the sheath was removed immediately after the operation and it was observed that the cumulative indwelling time was approximately equal to the catheter operation time. Therefore, it also showed that long-time catheter operation was a high-risk factor of radial artery occlusion. The longer the catheter operation time and the indwelling sheath time of the radial artery, the more serious the local injury and ischemia, the more prone to radial artery spasm and thrombosis, the aggravation of local repair and proliferation reaction, the active proliferation and migration of fibroblasts, and finally the radial artery occlusion [15–17]. Local thrombosis after radial artery injury is a high-risk factor for radial artery occlusion. The risk of radial artery occlusion [18–20] may be reduced intraoperatively or postoperatively by the use of anticoagulants and antiplatelet therapy.

Coronary heart disease and peripheral arterial disease are highly affected by diabetes [21, 22]. While diabetes causes coronary heart disease, it may also be associated with peripheral arterial radial atherosclerosis. Apart from oxidative stress, endothelial dysfunction, low-grade inflammation, and platelet hyperactivity, the vascular wall was affected by other metabolic abnormalities such as insulin resistance, hyperglycemia, and excessive release of free fatty acids in diabetes. Vasoconstriction and promotion of thrombus formation are further advanced by the motivation of these activities, eventually leading to the development of atherosclerosis [23]. Diabetic patients with impaired radial artery endothelial function may be more prone to spasm from endogenous vasoconstrictors [24]. Diabetic patients in addition have a higher incidence and severity of radial artery calcification than patients without diabetes [25]. 2 nondiabetic patients, the conclusion here indicated that the risk of right radial artery occlusion in diabetic patients was 2.186 times higher (95% CI (1.014–4.714), *p*=0.047). Atherosclerosis is also likely to be affected by elevated LDL cholesterol [26, 27]. Coronary heart disease patients complicated with hypercholesterolemia, on the one hand, may be complicated with radial arteriosclerosis stenosis. In addition, repeated radial artery injury will aggravate the speed of radial arteriosclerosis and cause chronic occlusion of the radial artery. The blood lipid data collected in this study are the blood lipid situation after taking statins for one year, which can reflect the real situation of blood lipid by long-term oral statins. The conclusion shows that poor low-density lipoprotein cholesterol control is a high-risk factor after coronary intervention for right radial artery occlusion (OR = 3.799, 95% CI (1.292∼11.166), *p*=0.015).

## 5. Conclusion

Diabetes, D-dimer elevation, low-density lipoprotein, cholesterol elevation, and long accumulated indwelling sheath time can easily cause radial artery occlusion.

Coronary heart disease and peripheral artery disease are highly affected by diabetes. Although diabetes causes coronary heart disease, it may also be associated with peripheral arterial radial atherosclerosis. The vascular wall, including oxidative stress, endothelial dysfunction, low-grade inflammation, and platelet overactivity, is influenced by other metabolic abnormalities such as insulin resistance, hyperglycemia, and excessive release of free fatty acids in diabetes. Cumulative indwelling sheath time is a predictor of radial artery occlusion. Therefore, diabetic patients should receive clinical attention. The duration of coronary intervention should be shortened as far as possible to reduce the time of indwelling sheath, full anticoagulation and antiplatelet during and after operation, and strict control of low-density lipoprotein cholesterol is likely to substantially decrease radial artery occlusion risks.

## Figures and Tables

**Figure 1:** Cumulative indwelling sheath time (hours) in the diagnosis of radial artery occlusion.

**Table 1:** Comparison of baseline data between the two groups.

	Not blocked (*n* = 449)	Block (*n* = 48)	Chi square/*Z*	*p*
Female	123 (27.4%)	18 (37.5%)	2.179	0.14
Age (years)^#^	64 (54∼71)	68 (52.5∼75.5)	−1.043	0.297
Body mass index (BMI)^#^	24.2 (20.5∼27.7)	25.25 (20.15∼28.75)	−0.677	0.498
Hypertension	220 (49%)	25 (52.1%)	0.165	0.684
Diabetes	86 (19.2%)	16 (33.3%)	5.345	0.021
Smoke	213 (47.4%)	20 (41.7%)	0.580	0.446
Hyperuricemia	20 (4.5%)	2 (4.2%)	0.008	0.927
D-dimer elevation	71 (15.8%)	16 (33.3%)	9.218	0.002
Acute coronary syndrome	235 (52.3%)	26 (54.2%)	0.058	0.809
Emergency percutaneous coronary intervention	113 (25.2%)	11 (22.9%)	0.117	0.732
Hypertriglyceridemia	115 (25.6%)	13 (27.1%)	0.049	0.825
Low HDL cholesterol	148 (33%)	17 (35.4%)	0.118	0.731
Elevated LDL cholesterol	21 (4.7%)	7 (14.6%)	8.004	0.005
Elevated serum lipoprotein a	104 (23.2%)	13 (27.1%)	0.370	0.543
Elevated serum creatinine	11 (2.4%)	2 (4.2%)	0.502	0.479
Elevated C-reactive protein	31 (6.9%)	4 (8.3%)	0.135^a^	0.713
Times of right radial artery route^#^	2 (2∼3)	3 (2.25∼3.75)	−4.493	<0.001
Accumulated indwelling sheath time (hours)^#^	2.1 (1.8∼2.6)	3.35 (2.8∼3.875)	−7.835	<0.001

*Note.* ^#^The nonnormal distribution obtained through the Shapiro–Wilk normality test, which is expressed by the median (lower quartile∼upper quartile).

**Table 2:** Multifactorial analysis of distal right radial artery occlusion.

		B	Standarderror	Wald	Freedom	Significance	OR	95% confidence interval of OR	
								Lowerlimit	Upperlimit
Diabetes	Yes	0.782	0.392	3.981	1	0.046	2.186	1.014	4.714
	No	0					1		
Elevated LDL cholesterol	Yes	1.335	0.55	5.885	1	0.015	3.799	1.292	11.166
	No	0					1		
D-dimer elevation	Yes	1.098	0.396	7.701	1	0.006	2.998	1.381	6.51
	No	0					1		
Accumulated indwelling sheath time (hours)		1.739	0.272	40.967	1	<0.001	5.692	3.342	9.694
Times of right radial artery route		0.006	0.267	0.001	1	0.981	1.006	0.596	1.699
Constant		−7.621	0.872	76.295	1	<0.001	0.001		

## Data Availability

The raw data supporting the conclusions of this article will be made available by the corresponding author, without undue reservation.
